RETRACTED

# A tree of life based on ninety-eight expressed genes conserved across diverse eukaryotic species

**DOI:** 10.1371/journal.pone.0184276

**Published:** 2017-09-18

**Authors:** Pawan Kumar Jayaswal, Vivek Dogra, Asheesh Shanker, Tilak Raj Sharma, Nagendra Kumar Singh

**Affiliations:** 1 National Research Centre on Plant Biotechnology, IARI, Pusa, New Delhi, India; 2 Banasthali University, Banasthali, Rajasthan, India; 3 Bioinformatics Programme, Centre for Biological Sciences, Central University of South Bihar, Patna, Bihar, India; National Institute of Plant Genome Research, INDIA

## Abstract

Rapid advances in DNA sequencing technologies have resulted in the accumulation of large data sets in the public domain, facilitating comparative studies to provide novel insights into the evolution of life. Phylogenetic studies across the eukaryotic taxa have been reported but on the basis of a limited number of genes. Here we present a genome-wide analysis across different plant, fungal, protist, and animal species, with reference to the 36,002 expressed genes of the rice genome. Our analysis revealed 9831 genes unique to rice and 98 genes conserved across all 49 eukaryotic species analysed. The 98 genes conserved across diverse eukaryotes mostly exhibited binding and catalytic activities and shared common sequence motifs; and hence appeared to have a common origin. The 98 conserved genes belonged to 22 functional gene families including 26S protease, actin, ADP–ribosylation factor, ATP synthase, casein kinase, DEAD-box protein, DnaK, elongation factor 2, glyceraldehyde 3-phosphate, phosphatase 2A, ras-related protein, Ser/Thr protein phosphatase family protein, tubulin, ubiquitin and others. The consensus Bayesian eukaryotic tree of life developed in this study demonstrated widely separated clades of plants, fungi, and animals. *Musa acuminata* provided an evolutionary link between monocotyledons and dicotyledons, and *Salpingoeca rosetta* provided an evolutionary link between fungi and animals, which indicating that protozoan species are close relatives of fungi and animals. The divergence times for 1176 species pairs were estimated accurately by integrating fossil information with synonymous substitution rates in the comprehensive set of 98 genes. The present study provides valuable insight into the evolution of eukaryotes.

## Introduction

Rapid advances in genome sequencing technology have added new dimensions to our understanding of the evolution of various species. The analysis of the gene contents of fully sequenced genomes has provided insights into the relationship between ecology and the genome evolution of different groups of flora and fauna [1]. The availability of large datasets such as unigenes and coding DNA sequences (CDSs) of different taxa in the public domain [e.g. National Centre for Biological Information (NCBI), DDBJ, ENSEMBL, and EMBL] has encouraged the analysis and functional characterisation of unique and conserved genes. The high-quality reference genomes of *Arabidopsis thaliana* [2] and *Oryza sativa* [3] have been extensively used as references for comparative analysis of plant genomes [4], and further extended to animals and microorganisms [5]. Currently, 3266 draft or reference genomes of eukaryotic species are available in the NCBI GenBank (https://www.ncbi.nlm.nih.gov/genome/browse/, accessed on 27 June 2016), of which 3173 have been categorised into 5 major groups: animal, fungus, plant, protist, and others. Fungi represent the largest number of sequenced eukaryotic genomes (n = 1609) in the public database, followed by animals (n = 900), protists (n = 375), and plants (n = 278). The large data set provides opportunities to compare multiple species and genera, facilitating the calibration of optimal evolutionary distances and identification of functionally conserved genes across species.

RETRACTED

The evolution of genes and genomes is driven by natural selection on genetic variations caused by the duplication, divergence, deletion, substitution, insertion, inversion, and translocation of DNA segments; of these, duplication and divergence are the most potent processes [6]. The duplication of genes, chromosomal segments, or the whole-genome, followed by neo-functionalisation, sub-functionalisation, and even pseudogenisation, contributes to the establishment of new gene functions underlying the origin of evolutionary novelty [7–9]. Comparative genomics is widely used for studying gene conservation between species and their evolutionary interrelationships [10, 11]. A single-copy gene-based analysis provided the evidence of the genome-wide conservation of synteny and co-linearity and clues to the origin of rice and wheat from a common ancestor [12]. The phylogenomics and synteny analyses of monocotyledonous and dicotyledonous plants have provided evidence for several rounds of whole-genome duplication [13, 14]. Synteny studies have used updated and dynamic approaches to understand cellular systems and processes among cereals to identify genes responsible for the basic cellular functions [15]. With the advent of next-generation sequencing (NGS) technology, large genomic sequence data have been deposited in the public domain and used for comparisons at a gene, gene network, or whole-genome level, and phylogenomics studies have illustrated the evolution of eukaryotic genomes [16, 17]. Different hypotheses and methodologies have been used to address the evolution of prokaryotic and eukaryotic genomes [18, 19].

RETRACTED

In this study, we performed a comparative analysis of expressed rice gene homologues in 48 other diverse eukaryotic species and developed a phylogenetic tree of life based on a comprehensive set of 98 genes conserved across these species. The fossil records of surviving and extinct species can aid in further confirming the accuracy of a phylogenetic tree. Therefore, we integrated the available fossil information with the DNA sequence data for developing the tree of life using the Bayesian approach.

## Materials and methods

### Model eukaryotic species and their sequence database

For the comparative genomics analysis, we used fully sequenced and annotated unigenes and the CDS sequences of 49 model species from different taxa of life such as plant, mammal, aves, reptile, amphibian, insect, and fungi as well as other lower animals. Among plants, we used data of the gymnosperms *Pinus taeda* and *Picea glauca* as well as some angiosperms; among angiosperms, we considered 7 monocotyledons, *Oryza sativa*, *Zea mays*, *Sorgham bicolor*, *Triticum aestivum*, *Hordeum vulgare*, *Brachypodium distachyon* and *Musa acuminata*, and 7 dicotyledons, *Arabidopsis thaliana*, *Cajanus cajan*, *Glycine max*, *Medicago truncatula*, *Solanum lycopersicum*, *Vitis vinifera*, and *Populus trichocarpa*. In addition, we considered lower plants such as the bryophyte, *Physcomitrella patens*, and a single-cell green alga, *Chlamydomonas reinhardtii*. Among the Animalia class, we included the data of 6 mammals, *Bos tourus*, *Homo sapiens*, *Mus Musculus*, *Pan troglodytes*, *Gorilla gorilla*, *Pongo abelii*, as well as a bird, *Gallus gallus*, an amphibian, *Xenopus laevis*, and a fish, *Danio reio*. Furthermore, we included 2 reptiles (*Anolis caroliensis* and *Pelodiscus sinensis*), 4 insects (*Drosophila melanogaster*, *Anopheles gambiae*, *Apis mellifera*, and *Bombyx mori*), and other lower animals—*Ciona intestinalis*, *Nematostella vectensis*, *Hydra magnipapillata*, *Strongylocentrotus purpuratus*, and *Caenorhabditis elegans* (round worm). For better representation of life in the model organism, we also included 7 fungi from the Ascomycota (*Aspergillus oryzae*, *Fusarium oxysporum*, *Neurospora crassa*, and *Magnaporthe grisea*), Basidiomycota (*Puccinia graminis* and *Cryptococcus gattii*) and Mucormycotina (*Rhizopus oryzae*). We also included 4 protist species, namely *Salpingoeca*, *Phytophthora*, *Dictyostelium* and *Toxoplasma* shown in Table 1. The data on all these species were downloaded from NCBI (http://www.ncbi.nlm.nih.gov/unigene), Broad Institute of Microbial Genome (https://www.broadinstitute.org/scientific-community/data), and Ensembl (http://asia.ensembl.org/index.html) databases. For constructing the tree of life, the aforementioned organisms were selected because they cover the widest range of species having the maximum number of expressed sequence tag (EST) and cDNA sequences (plants ≥ 10 500, animals ≥ 2000, and algae/fungi ≥ 10000).

RETRACTED

**Table 1:** Information of 49 selected model organism for the comparative genomic analysis.

	Kingdom/Phylum	Sub Category (Scientific Name)	Genome Size (MB)	EST Unigene /CDS /cDNA
**A**	Kingdom Plantae			
	Eudicotyledons	*Arabidopsis thaliana*	125	30633*
		*Cajanus cajan*	858	59,515
		*Glycine max*	1,115	35982*
		*Medicago truncatula*	390	18045*
		*Populus trichocarpa*	485	15056*
		*Solanum lycopersicum*	900	18071*
		*Vitis vinifera*	487	22501*
	Liliopsida	*Brachypodium distachyon*	272	10698*
		*Oryza sativa*	389	44235*
		*Zea mays*	2,500	92266*
		*Triticum aestivum*	17,000	56955*
		*Hordeum vulgare*	5,100	26945*
		*Sorgham bicolor*	772	13736*
	Zingiberales	*Musa acuminata*	523	36549^◊^
	Chlorophyta	*Chlamydomonas reinhardtii*	121	7579*
	Streptophyta	*Physcomitrella patens*	487	17573*
	Gymnosperm	*Pinus taeda*	20,100	17390*
		*Picea glauca*	20,000	27848*
**B**	Kingdom Fungi & Protista			
	Ascomycota	*Aspergillus oryzae*	37	12,063^†^
		*Fusarium oxysporum*	59.9	17,708^†^
		*Neurospora crassa*	39.9	17,073*
	Basidiomycota	*Puccinia graminis*	89	15,979^†^
	Mucormycotina	*Rhizopus oryzae*	45.3	17459^†^
		*Magnaporthe grisea*	40.3	11054^†^
		*Cryptococcus gattii*	18.4	6,210
	Oomycetes	*Phytophthora infestans*	240	8920*
	Apicomlexa	*Toxoplasma gondii*	63	6237*
	Dictyosteliida	*Dictyostelium discoideum*	34	6187*
	Chytridiomycota	*Salpingoeca rosetta*	55	11736^†^
**C**	Kingdom Animalia			
	Mammalia	*Bos tourus*	2,860	45364*
		*Homo sapiens*	2,910	130055*
		*Mus Musculus*	2,500	30386*
		*Pan troglodytes*	2,400	20479●
		*Gorilla gorilla*	3035	29026●
		*Pongo abelii*	3,080	22451●
	Reptiles	*Pelodiscus sinensis*	2,200	20765●
		*Anolis caroliensis*	1,780	25137*
	Actinopterygii	*Danio reio*	1,412	53559*
	Amphibia	*Xenopus laevis*	3,000	31434*
	Ascidiacea	*Ciona intestinalis*	160	28121*
	Aves	*Gallus gallus*	1,050	34025*
	Echinodermata	*Strongylocentrotus purpuratus*	814	14718*
	Insecta	*Apis mellifera*	1,800	24392*
		*Drosophila melanogaster*	180	17132*
		*Bombyx mori*	530	13952*
		*Anopheles gambiae*	278	14672*
	Nematoda	*Caenorhabditis elegans*	97	23151*
	Cnidaria- Anthrozoa	*Nematostella vectensis*	450	14574*
	Cnidaria-Hydrozoa	*Hydra magnipapillata*	1,000	11072*

*unigene: https://www.ncbi.nlm.nih.gov/unigene

◊cds:http://banana-genome.cirad.fr/download

†: https://www.broadinstitute.org/fungal-genome-initiative

●cDNA:http://asia.ensembl.org/index.html

RETRACTED

### Identification of rice gene homologues in other eukaryotic species

To identify the homologous gene sequences among 49 model organisms we have downloaded 66338 CDS (90.57 MB) and 44235 EST-unigene sequences (72.86MB) from the fully sequenced and annotated genome of *O*. *sativa* from the Rice Genome Annotation Project Database (http://rice.plantbiology.msu.edu/) and NCBI (ftp://ftp.ncbi.nlm.nih.gov/repository/UniGene/Oryza_sativa/), respectively. To identify the uniquely expressed rice genes, we used a locally configured BLASTN [20] programme with pre-optimised blast parameter [21], in which unigenes and CDS sequences were treated as query and subject, respectively, was used. In this process, we identified the chromosomal position of 44235 EST-unigene sequences; after removing the splicing sites from the expressed sequence, 36002 EST-unigenes were considered for further comparative analysis. The top hit on the subject genome was retrieved using Blast Parser (version 1.2.6.14) [22], with ≥300 bit score and ≥60% sequence identity. The extracted homologous sequences was used as a query, whereas 48 other model organism sequences used as a subject, with ≥100 bit score and ≥60% sequence identity. All matched homologous gene sequences of the 48 model species were distributed with respect to the 12 chromosomes of rice by using a Microsoft Excel-based programme. The Blast2GO tool [23] was used for the functional annotation of the rice gene. The details are presented in a flowchart (Fig 1).

**Fig 1:** Pipeline to identify and analyse the conserved gene among 49 species and development of phylogenetic tree. Flow diagram showing scheme of genome wide comparative analysis of rice genes in 48 other eukaryotic species.

### Bayesian analysis of origin of 98 rice genes conserved across eukaryotes

Bayesian inferences (BIs) were detected for the starting tree of 98 conserved rice gene sequences with Mrbayes (version 3.2.2) [24]. We used 3 partitions, and the analysis comprised 50 million generations, with a sample frequency of 100 generations and a standard deviation value of 0.01. First 25% of the total run was discarded as burn-in. The phylogenetic tree was visualised using Figtree (version 1.4.0) [25]. The alignment obtained using the default settings in mafft-7.047-win64 [26] is available from TreeBase (http://purl.org/phylo/treebase/phylows/study/TB2:S20689).

### Development of the phylogenetic tree of 49 model eukaryotic species

The phylogenetic tree analyses were performed using 2 separate methods—Maximum Likelihood (ML) and BI. The ML analysis was implemented using MEGA 5 [27]. Statistical reliability for individual node support was determined from the 1000 replicates of a non-parametric bootstrap with 5 discrete gamma categories and the initial developed tree was supported using the neighbour-joining method [28]. The best-fit substitution model for each codon and gene was identified using a 24 nucleotide substitution model on MEGA 5. On the basis of the BI criterion, we selected the best-fit substitution model [general time-reversible (GTR) + discrete gamma distribution (G) + evolutionary invariable (I)]. The analysis included 98 conserved gene sequences among 49 organisms and 1st+2nd+3rd+noncoding codon positions. All positions containing gaps and missing data were eliminated, and the total number of positions was 84544 in the final data set. The BI analysis was performed using Mrbayes (version 3.2.2), with 2 initial independent runs conducted for 5000000 generations, saving trees every 100 generations. A reversible jump Markov chain Monte Carlo (RJ-MCMC) substitution scheme was used with a discrete gamma distribution model and 6 substitution types during the run. Three partitioning strategies were used, and the defined model parameters unlinked between partitions. In both phylogenetic trees, *C*. *reinhardtii* was considered as the outgroup. The output of Mrbayes was examined using Figtree (version 1.4.0) and Tracer (version 1.6) [29]. All identified conserved homologous gene sequences among the 49 species were concatenated and aligned using edit plus 3 and mafft-7.047-win64 respectively. The aligned file is available from TreeBase (http://purl.org/phylo/treebase/phylows/study/TB2:S20689).

RETRACTED

### Estimation of evolutionary divergence time between species

Divergence time was estimated among the 98 conserved gene sequences of 49 model species. For the synonymous substitution values (Ks), a total of 115248 pairwise combinations were formed using the formula {(n × (n-1))/2} × 98, where n is the number of species. We estimated the synonymous substitution rate (r) values for all combinations according to the method by Nei and Gojobori [30] implemented in DnaSP (version 5.0) [31]. The calculated Ks values were tabulated in 3 statistical categories, namely mode, median, and average, and the molecular clock was estimated using the formula r = Ks/2T, where r is the number of substitution per site per year and T is the divergence time (in million years) between 2 sequences. Simultaneously, BEAST (version 1.8.0) [32] was used for the estimation of divergence time and the phylogenetic analyses were conducted using the MCMC method. The BEAST analysis was performed using the substitution model, GTR heterogeneity model, with gamma (G) plus invariable (I), from which the r parameters and base frequencies across the codon positions were unlinked. An uncorrelated lognormal relaxed-clock model was used, with the birth–death process as a tree prior. The uniform distribution value was used as the relative rate parameter for codon positions 1, 2, and 3. Our estimates for the origin of the 49 eukaryote model organism were based on fossil treatments. All sampled species were grouped into 6 categories lower plants (*C*. *reinhardtii* and *P*. *patens*), angiosperms (*O*. *sativa*, *T*. *aestivum*, *Z*. *mays*, *H*. *vulgare*, *M*. *acuminata*, *S*. *bicolor*, *B*. *distachyon*, *G*. *max*, *V*. *venifera*, *C*. *cajan*, *A*. *thaliana*, *M*. *truncatula*, *S*. *lycopersicum*, *and P*. *trichopara*), gymnosperms (*P*. *taeda* and *P*. *glauca*), fungi (*A*. *oryzae*, *F*. *oxysporum*, *N*. *crassa*, *P*. *graminis*, *R*. *oryzae*, *M*. *grisea*, *and C*. *gatti*), vertebrates (*B*. *torus*, *H*. *sapiens*, *M*. *musculus*, *G*. *gorilla*, *P*. *troglodytes*, *P*. *abelii*, *D*. *rerio*, *X*. *laevis*, *G*. *gallus*, *P*. *sinensis*, and *A*. *carolinensis*), and invertebrates (*C*. *elegans*, *C*. *intestinalis*, *H*. *magnipapillata*, *N*. *vectensis*, and *S*. *purpuratus*). We used the following fossil information for all 49 species and grouped them into 6 separate categories: 1500 million years ago (Ma) [33], 132 Ma [34, 35], 270 Ma [36, 37], 438 Ma [38], 365 Ma [39], and 750 Ma [40]. The concatenated aligned sequences of the 98 conserved eukaryotic genes were analysed in 3 independent runs between 200 and 1000 Ma, following a 10% burn-in in each run. The convergence of the chain to stationary distribution was ensured by combining all 3 independently generated log files by using Tracer. More than 2000 million states were analysed, and the estimated sample size (ESS) for all 6 groups was in the range of 1321–405700, whereas the posterior and prior were 113 and 334, respectively.

RETRACTED

## Results

### Genes expressed uniquely in rice

Despite having a common ancestor, different species have evolved various unique traits and functions. Notably, we observed that of the total 36002 EST-unigenes expressed in rice, 9831 (27.3%) are unique. The remaining 26171 genes (72.7%) matched substantially with one or more of the 48 other analysed eukaryotic species. The 9831 unique rice genes are distributed on all the 12 rice chromosomes, but the highest number of 1019 such genes is located on chromosome 4, followed by 977 genes on chromosome 1. The lowest number of genes (n = 649) is on chromosomes 9 and 10 (Figure A in S1 File). However, these numbers are partly confounded by the size of the rice chromosomes; the highest proportion of unique rice genes to the total number of expressed genes is on rice chromosome 12 (36.02%), followed by chromosome 11 (34.49%; Figure Ab in S1 File).

To understand the functional annotations of the 9831 unique rice genes we performed gene ontology (GO) based automated annotation using the Blast2GO programme, which identifies protein domains in the gene sequence by using BLASTX matches in the NCBI non-redundant database. Among all unique rice genes, a 7267-protein model was GO-annotated, whereas another 2564-protein model did not demonstrate any significant GO match in the database (Figure B in S1 File). The classification of 7267 GO-annotated genes on the basis of their biological process, cellular localisation, and molecular function indicated that the maximum number of genes belongs to the metabolic (n = 3759) and cellular (n = 2757) processes, organelle (n = 4473) and cell (n = 4521) categories, and binding (n = 4199) and catalytic (n = 3636) activities, respectively. The BLAST search-based annotation of the 9831 unique rice genes revealed that the largest category is transposable element (TE)-related genes (n = 6313, 64.21%; Fig 2; Table A in S2 File). However, the second largest category of unique rice genes (n = 2388; 24.29%) has unknown function. The other large families of unique rice genes with known function were as follows: F-box domain containing proteins (n = 177), 122 genes with disease resistance and defence response-like proteins (n = 122), zinc finger proteins (n = 106), protein kinases (n = 52), seed storage proteins (n = 38), no apical meristem family proteins (n = 24), and pollen allergen family proteins (n = 20). Furthermore, among the 9831 uniquely expressed rice genes, 7614 (77.44%) have an intron, whereas the remaining 2217 (22.55%) do not, with an average number of 3.08 introns per gene and 1.01 introns per kbp (Table B in S2 File).

**Fig 2:** Annotation of uniquely expressed genes in rice. Functional annotations of 9,831 genes uniquely expressed in rice in comparison to 48 other eukaryotic species. Annotations with more than ten genes per family only are shown here.

### Expressed rice gene homologues in other plant species

A comparative analysis of expressed rice gene homologues in 17 other plant species revealed crucial information regarding the evolution of the Poaceae and other plant families. Regarding the Poaceae family members, 9948 (27.63%) genes are expressed commonly in all the 5 species (*T*. *aestivum*, *Z*. *mays*, *H*. *vulgare*, *S*. *bicolor*, and *B*. *distachyon*). *Z*. *mays* shows the highest number of matches with 22305 expressed rice genes, closely followed by *H*. *vulgare* (n = 21700) and *T*. *aestivum* (n = 21059). Of the 9948 genes conserved in the Poaceae family, rice chromosomes 1 and 3 show the highest number of matches (n = 1911 and 1736, respectively), whereas chromosomes 11 and 10 show the lowest number of matches (n = 663 and 708, respectively; Fig 3). Among other plant species, *A*. *thaliana* share 11321 (31.44%) expressed genes with rice. Three legume species have a matching of 27.8%–39.5% of the rice genes, with *C*. *cajan* sharing the maximum number of genes (n = 14230), followed by *G*. *max* (n = 12663) and *M*. *truncatula* (n = 9993). Two gymnosperm species, *P*. *taeda* (southern yellow pine) and *P*. *glauca* (white spruce) demonstrate 7124 (19.79%) and 9930 (27.58%) matches, respectively (Fig 3). We also compared the 36002 rice EST-unigene sequences with bryophyte monoecious moss *P*. *patens* and observed 6187 (17.18%) rice gene homologues. Of the 36002 expressed rice genes, 2841 (7.89%) were commonly expressed in all 17 plant species and 9838 (27.32%) were uniquely expressed in rice. The annotation of the 2841 conserved genes among all 17 plant species indicated that many plant cellular component genes responsible for respiration, photosynthesis, photomorphogenesis, growth, and development are conserved and that most of them were located on rice chromosomes 1 and 3 (Fig 3; Figure C in S1 File, Table C in S2 File). The frequency distribution of the 2841 conserved genes indicated that most of the genes from the protein kinase, phosphatase, transferase, dehydrogenase, and ribosomal protein families shared more than 103 genes in each family (Figure C in S1 File). However, in the context of unique rice genes, only 59 genes have unknown function and 29 genes code transposon proteins.

RETRACTED

**Fig 3:** Clustering of homologs genes in between rice and other plant species. Chromosome wise distribution of expressed rice gene homologs expressed in 16 other plant species. Parenthesis showed the number of homologs gene of individual species.

### Expressed rice genes homologues in fungal and protist species

Chromosome wise number of expressed rice gene homologues present in 7 fungal and 4 protist species in shown in Table 2. Among the 7 analysed fungal species, *R*. *oryzae*, has the highest number of 1179 expressed rice gene homologues, followed by *M*. *grisea* (n = 752); by contrast, *P*. *graminis* has the lowest number of rice gene homologues (n = 593). Among all fungal species, *C*. *gattii* has the highest proportion of rice gene homologues (10%), whereas the remaining 6 have a matching of 3.71%–6.8% of the total genes (Table 2). Our analysis revealed that 313 rice gene homologues are conserved among all 7 fungal species, distributed in all 12 rice chromosomes. The highest number of genes is on chromosome 1 (n = 54), followed by chromosome 3 (n = 52), whereas chromosome 12 shows the lowest number of matching genes (n = 9; Figure D in S1 File). Most of the 313 annotated rice gene homologues, conserved across fungal species, tend to support the basic cellular and metabolic functions (Figure E in S1 File). Genes coding ribosomal proteins, protein kinase, histone, ubiquitin, DnaK, ras-related proteins, tubulin, 26S protease, phosphatase actin, and DEAD-box proteins have more than 10 matches per gene family, whereas the dehydrogenase family shows 9 matches. Other essential genes conserved between rice and all 7 fungi include heat shock protein (Hsp70/Dnak), which are involved in abiotic stress tolerance.

RETRACTED

**Table 2:** Frequency distribution of expressed rice gene homologs in seven different fungal and four protista species. The number shown in the column represent the distribution of the expressed homologous rice gene sequences among the total unigene of their respective organisms.

Fungus and Protista species	Total no. of genes	Number of conserved genes on rice chromosome												
		Chr1	Chr2	Chr3	Chr4	Chr5	Chr6	Chr7	Chr8	Chr9	Chr10	Chr11	Chr12	Total
*R*. *oryzae*	17459	142	116	152	95	116	93	99	81	68	72	67	78	1179
*M*. *grisea*	11054	96	92	114	58	87	72	52	44	34	34	34	35	752
*F*. *oxysporum*	17708	108	83	111	46	84	69	58	43	36	32	36	40	746
*A*. *oryzae*	12063	106	83	113	39	85	59	56	42	33	31	30	37	714
*N*. *crassa*	17073	103	73	108	45	80	62	48	37	34	28	29	34	681
*C*. *gattii*	6210	101	78	105	36	76	56	53	33	32	30	29	34	663
*P*. *graminis*	15979	88	74	98	31	63	54	47	29	24	31	25	29	593
*P*. *infestans*	8920	194	165	187	91	131	102	92	74	61	59	52	58	1266
*S*. *rosetta*	11736	116	109	127	46	86	75	58	47	47	33	41	44	829
*T*. *gondii*	6237	83	65	87	29	66	51	40	27	32	29	28	28	565
*D*. *discoideum*	6187	73	60	82	32	48	44	32	25	20	24	23	24	487

Among all 4 analysed protist species, *P*. *infestans*, the causative agent of late blight in potato, shows the highest number of matches with rice gene homologues (n = 1266), followed by unicellular choanoflagellate species, namely *S*. *rosetta* (n = 829) and *T*. *gondii* (n = 565), and finally, *D*. *discoideum* (n = 487) from the phylum Amoebozoa. In all 4 protist species, 238 rice gene homologues were conserved; these were distributed on all 12 rice chromosomes (Figure F in S1 File). These 238 conserved genes were classified into 40 functional categories with more than 13 genes in each category (Figure G in S1 File), the major groups were as follows: ribosomal proteins, protein kinases, ubiquitin, 26S protease regulatory proteins, DnaK and ras-related proteins, with more than 13 genes in each category (Figure G in S1 File).

RETRACTED

### Expressed rice gene homologues in animal species

We searched for the presence of 36002 expressed rice gene homologues in 20 animal species belonging to both higher and lower levels of the animal kingdom—11 vertebrates and 9 invertebrates. The highest number of matches between rice and animal species were observed in 6 mammals—*H*. *sapiens* share the highest number of rice gene homologues (n = 1222), followed by *B*. *torus* (n = 1076) and *M*. *musculus* (n = 1057; Figure G in S1 File). Two reptiles, *P*. *sinensis* (soft shell turtle) and *A*. *carolinensis* (green anole) share 1000 and 776 rice gene homologues, respectively. Similarly, one each of fish, amphibian, and bird species share 1056, 994, and 988 rice gene homologues, respectively (Figure G in S1 File). Among the nine invertebrates, *H*. *magnipapillata* and *N*. *vectensis* (small sea anemone) shared the lowest (n = 618) and the highest (n = 903) number of rice gene homologues, respectively (Figure G in S1 File). Four insect species, *A*. *mellifera*, *D*. *melanogaster*, *B*. *mori*, and *A*. *gambiae*, share 700–862 rice gene homologues. Similar to the gene distribution in the plant species, the conserved rice gene homologues in different animal species are distributed on all 12 rice chromosomes (Fig 4). We observed that 154 expressed rice gene homologues, belonging to 30 functional categories, are conserved among all 20 analysed animal species (Figure H in S1 File). These conserved rice gene homologues include the heat shock protein, 26S protease regulatory subunit, tubulin, phosphatase, protein kinase, and actin, which contain more than 10 genes in each family. Six genes encode the DEAD-box RNA helicase family proteins, responsible for nuclear export, translation initiation, pre-mRNA splicing [41, 42]. The comparison of rice genes with those of nine invertebrate species showed that the 195 rice gene homologues are specifically expressed in invertebrate species and that all these belong to 43 gene families. Most of the conserved genes are protein kinases, heat shock proteins, 26S proteasomes, tubulins, phosphatase 2A (PP2A), actin, ras-related proteins, ATP-dependant RNA helicase, and dehydrogenase family proteins, with more than 10 genes in each family (Table D in S2 File). Notably, of the 195 conserved genes, 24 are uniquely expressed in only the 9 invertebrate species among the 20 animals. For instance, 8 rice gene homologues are of glycogen synthase kinase and 3 of cyclin-dependant kinase, which are broadly responsible for the abscisic acid stimulus and cell cycle control, respectively, are uniquely expressed in the invertebrate species (Table E in S2 File). Other rice genes, such as those encoding pre-mRNA-processing-splicing factor, ribonucleoside-diphosphate reductase, and signal recognition particle, are conserved among invertebrate species.

RETRACTED

**Fig 4:** Clustering of homologs genes in between rice and animal species. Chromosome wise distribution of rice gene homologs expressed in 20 different animal species. Figures in parenthesis indicate total number of EST-unigenes in the respective animal species.

We compared of the rice genes with that of 11 vertebrate species and observed that several gene homologues are expressed in specific vertebrate species. In total, 413 rice gene homologues belonging to 82 functional categories are commonly expressed in all 11 vertebrate species; some genes, such as ribosomal proteins L3/L5/L13/L22 and S2, are expressed in mammals as well as other vertebrate species (Table F in S2 File). Categorically, 6 copies of the 14-3-3 protein rice homologue, which plays a crucial role in various regulatory processes including apoptotic cell death, cell cycle control, and mitogenic signal transduction, are conserved in all the vertebrate species. Similarly, 5 rice gene homologues of fructose bisphosphate aldolase isozyme, expressed in the muscles, liver, and brain of mammals, are conserved among all the vertebrate species. The PINHEAD genes responsible for the formation of primary axillary shoot apical meristems, as reported in *Arabidopsis*, are present in rice as well as all 11 vertebrate species. Other examples of expressed rice gene homologue in vertebrates include calreticulin precursor, cell division cycle protein, coatomer subunit beta-1/gamma-2, and puromycin-sensitive amino peptidase protein (Table F in S2 File). A set of 30 single-copy genes is present in all 11 vertebrates.

In total, 727 rice gene homologues are conserved and expressed in all 6 analysed mammalian species. The annotation of these conserved genes could be classified into 156 functional categories. Of these, 524 genes belong to 35 major families, each with 5 or more genes (Figure I in S1 File), whereas the remaining 203 genes belong to 121 families. The largest gene families commonly expressed in rice and all the 6 mammalian species include ribosomal proteins (n = 68), protein kinase (n = 57), core histones (H2A, H2B, H3, and H4; n = 42), ras-related proteins (n = 39), and ubiquitin domain-containing proteins (n = 30), which play crucial roles in protein translation, phosphorylation, DNA packaging, signal transduction, and apoptosis, respectively.

### Expressed rice genes conserved across eukaryotes and their evolution

The genome-wide analysis of expressed rice gene homologues in 48 diverse eukaryotic species identified 98 genes conserved across all these species (Table G in S2 File). The comprehensive set of conserved genes are distributed on all 12 rice chromosomes with chromosomes 1–3 collectively carrying more than 50% of the conserved genes, in contrast to the density of unique rice genes, which is the highest on chromosomes 11 and 12 (Figure Ab in S1 File). The 98 conserved genes belong to 5 broad functional categories: nucleic acid metabolism, protein metabolism, physiological functions, transportation, and stress response. The GO-based annotation of the 98 genes grouped them based on the major criteria of biological process, cellular localisation, and molecular function (Fig 5A–5C). According to the biological process, the 4 largest categories of genes are those encoding the constituents of cellular processes (18.35%), metabolic processes (16.22%), single organism processes (14.63%), and response to stimulus (14.10%), with 10 other minor categories including reproductive, cellular component organisation, developmental process, biological regulation, growth, multiorganism processes, biological phase, localisation, multicellular organismal processes, and signalling. On the basis of the cellular localisation criteria, the major categories encode cells (29.41%), organelles (24.84%), membranes (20.26%), macromolecular complexes (12.09%), and membrane-enclosed lumens (7.84%). On the basis of the molecular functions, genes encoding binding nature proteins (48.57%) and catalytic activities (37.71%) are the most abundant categories. Furthermore, the observed intron density (5.97 per gene, 1.49 per kbp) in the 98 conserved genes is significantly higher than that of the unique in rice genes (3.08 per gene, 1.01 per kbp; Table H and B in S2 File).

RETRACTED

**Fig 5:** Gene annotation. Gene ontology (GO) based annotation of 98 rice genes conserved across 49 eukaryotic species using BLAST2GO programme. The genes were classified based on three different criteria: (a) Biological process, (b) Cellular localization and (c) Molecular function.

On the basis of their annotated functions (Table G in S2 File), the 98 conserved genes belong to 22 gene families. The largest families encode the DnaK chaperone protein (n = 12), actin (n = 10), 26S proteasome subunits containing multicatalytic threonine proteases (n = 10), tubulin (n = 9), DEAD-box protein (n = 6), serine/threonine protein phosphatase (n = 6), and ubiquitin protease (n = 6). Furthermore, 5 genes encode PP2A, playing a critical role in the regulation of signal transduction in a cell. ADP-ribosylation factor and ras-related protein, both of which belong to the Ras superfamily that is involved in posttranslational modification as well as transmitting signals within the cell, are represented by 5 and 3 genes, respectively. Four genes each for ATP synthase and glyceraldehyde 3-phosphate dehydrogenase are also conserved among all 49 species. The casein kinase I and II gene families, which also encode serine/threonine protein kinases, are conserved in 3 and 1 gene, respectively. Three genes each were observed for enolase enzymes responsible for the glycolysis or fermentation and elongation factor for protein translation were observed. Two conserved families with 2 genes each (cell division control protein and calmodulin) and 5 conserved families with 1 gene each (oligosaccharyl transferase, succinate dehydrogenase, flavoprotein, T-complex protein and an unknown protein) were also observed.

Because these 98 genes are conserved across the entire range of lower and higher eukaryotes, they must be highly essential for the evolution of early eukaryotes. To explore their interrelationship, we compared these 98 EST-unigenes of rice by using multiple sequence alignments and constructed a Bayesian phylogenetic tree. A significant level of sequence conservation (Fig 6A and 6B) was observed. Furthermore, a high level of sequence conservation is present among different genes with the same annotated function (e.g. actin, DnaK, ubiquitin, tubulin, and PP2A genes), which are grouped together in the phylogenetic tree (Fig 6A). Notably, significant conservation of sequence motifs can be present between genes belonging to different functional categories (Fig 6B and Figure J in S1 File). The results of the statistical analysis of the phylogenetic tree revealed ESS of 3746.09 of total tree length and a potential scale reduction factor of 1.000051, suggesting a strong support for the node clusters (Table I in S2 File). The presence of conserved sequence motifs among the 98 rice genes with different functional categories suggests that they may have originated from common ancestral genes during the evolution of early eukaryotes. ADP-ribosylation factor and elongation factor, both of which participate in the protein translation process in both prokaryotes and eukaryotes, are grouped together at the base of the phylogenetic tree. Nine tubulin domains containing proteins form a single clade with 6 ubiquitin genes with a posterior probability (PP) of 1.0, demonstrating strong node formation between the groups. Similarly, 4 casein kinase genes form a single clade with 6 serine/threonine protein phosphatase and PP2A genes, as these belong to the same protein kinase group and play a crucial role in signal transduction [43].

RETRACTED

**Fig 6:** Phylogenetic tree of conserved gene sequences of *Oryza sativa*. **(a)** Phylogenetic tree of 98 expressed rice gene homologs conserved across 49 eukaryotic species. Unrooted Bayesian tree was constructed after alignment of the 98 rice CDS sequences. Posterior probability of each clade is shown at the respective node. **(b)** Multiple sequence alignment of 22 of the 98 rice genes, taking one representative from each functional category. Nucleotide base is color coded to facilitate visualization of the homology. The Jalview alignment picture was cropped to show the conserved parts of the genes. Black bars at the bottom show the level of sequence conservation.

### A tree of life based on 98 genes conserved across eukaryotes

We constructed phylogenetic trees of life for the 49 eukaryotic species, including rice, based on the 98 conserved genes by using ML and BI methods. The 98 EST-unigene sequences for each species were first concatenated to create a composite-gene sequence. The aligned composite gene sequences of the 49 species were analysed and *C*. *reinhardtii*, the most common ancestor of plant and animal species, was selected as the outgroup. In the ML tree, the level of uncertainty for the node formation is high and specifically to the selected insect and fungal species (Figure K in S1 File). Therefore, to achieve a highly robust grouping of the 49 species, we developed a Bayesian phylogenetic tree by using Mrbayes (Fig 7), with a more robust node support than the variable bootstrap values observed for the ML tree. The summarised sampled parameters (.p) file shows average ESS of more than 200 (13356.74–133937.4244) and a potential scale reduction factor of nearly 1.0 (0.9999–1.0000; Table J in S2 File). Our Bayesian phylogenetic tree is well resolved with a PP of 1.0 for almost all nodes, except the 3 for fungal species *P*. *graminis*, *C*. *gatti*, and *R*. *oryzae*, which have lower PPs of 0.5 (Fig 7). In the eukaryotic tree, the 49 species were clustered into 2 broad groups of plants and animals. The fungi grouped with animals as a separate sub-clade and; the 4 protist species are placed with their closest plant, animal, or fungal clade. The 17 plant species were grouped into 3 clusters of angiosperms (14 species), gymnosperm (2 species), and bryophyte (1 species). Furthermore, the 14 angiosperms were subcategorized into 2 broad classes of monocotyledons and dicotyledons with banana (*M*. *acuminata*), showing a link between the 2 classes. In the monocotyledon clade, *Triticum*, *Hordeum*, and *Brachypodium* were significantly diverged from *Oryza* and had a common origin point along with *Zea* and *Sorghum*. In dicotyledonous species, 3 closely related legume genera, *Glycine*, *Cajanus*, and *Medicago*, formed a single clade. *Vitis–Populus* and *Arabidopsis–Solanum* are distantly related and formed separate clades. *Physcomitrella* is the outermost clade among the 17 plant species. In the phylogenic tree, 20 animal species, including mammals, reptiles, birds, amphibians, fishes, and insects, formed an expected monophyletic clade. Among the 6 mammals, mice were closer to the base of the tree and are most closely related to cow, which in turn, is closer to primates than to mice. By contrast, among the 4 primates, humans are most closely related to chimpanzees. Our Bayesian tree showed that chimpanzees, gorillas, and orangutans form a single clade. Two reptile species, *Anolis* and *Pelodiscus*, are grouped along with the bird *Gallus*, followed by amphibian and fish. In the invertebrate clade, 4 insect species form a clear single cluster: *A*. *mellifera* (honey bee) was grouped closer to *B*. *mori* (silkworm), whereas *D*. *melanogaster* (fruit fly) and *Anopheles* (mosquito) formed a separate clade. The 7 fungal species were clearly differentiate into 3 phyla, namely Ascomycota, Basidiomycota, and Mucormycotina. Our results demonstrated that *S*. *rosetta*, a choanoflagellate protists closely related to animals, establish a link between animal and fungi, whereas another protist *D*. *discoideum* from the Amoebozoa phylum is located as an outer group of fungal species. Two other protist species, *P*. *infestans* and *T*. *gondii*, are closer to *C*. *reinhardtii*, which itself is a unicellular green algae located as an outermost group in the Bayesian tree. Overall, the 98 gene based phylogenetic tree is consistent with a larger dataset and as such impress our understanding of the evolution of plants, fungi and animals.

RETRACTED

**Fig 7:** Eukaryotic tree of life. A rooted eukaryotic phylogenetic tree based on concatenated sequences of 98 rice gene homologs conserved across 49 eukaryotic species using Bayesian approach (Mrbayes v 3.2). Bayesian posterior probability for each node is 1. Tree was rooted using *Chlamydomonas reinhardtii* (Green algae) sequence.

### Divergence time of eukaryotic species based on synonymous substitution rates

Synonymous substitution rates are frequently used to estimate the time of divergence for a pair of species based on the evolutionary clock assuming a uniform rate of spontaneous mutations at the synonymous single-nucleotide polymorphism positions. To explore the divergence times of the 49 species, we estimated the synonymous substitution values (Ks) in pairwise combinations of species for the 98 conserved genes, requiring 115248 gene pairs [(49×48)/2 × 98] of sequence alignments (Table K in S2 File). Next, we analysed data to decide whether to consider the mean, median, or modal Ks values of the 98 genes for estimating overall synonymous substitution rate (r) and divergence time for the 1176 pairwise combinations of species: A representative sample of 50 pairs of the 1176 pairwise combinations is presented here for this comparison. For each of the 50 pairs, 10 frequency distribution graphs of randomly selected genes—10 genes, 4 graphs; 20 genes, 3 graphs; 40 genes, 2 graphs; and all genes, 1 graph—were plotted. These conserved genes had low modal Ks values, lying invariably in the first interval between 0 and 0.1. Therefore, instead using the of earlier reported modal Ks values for the estimation of divergence times between species, we used mean Ks values for estimating the r values as suggested by Graur and Li [44] and median Ks values for estimating species divergence time [45]. The result of the 50 representative pairs is shown in Table 3, and a complete list of 1176 pairs is provided in Table L in S2 File. Among the 6 monocotyledonous species, we observed the lowest mean Ks value of 0.13 between *T*. *aestivum* and *H*. *vulgare*, which are closely related to each other, whereas the distantly related monocotyledonous species *Z*. *mays* and *M*. *acuminata* showed the highest Ks value of 0.69. For estimating divergence times, we first calculated the r values using the mean Ks values, followed by the divergence times in Ma by using the median Ks values, calculated using the molecular clock of Muse and Weir [46] and calibration times based on the published fossil information (Table 3; Table L in S2 File), e.g. 110 Ma for angiosperms, [35]). These values indicate that closely related cereal crop pairs *Z*. *mays*–*S*. *bicolor* and *T*. *aestivum*–*H*. *vulgare* diverged from each other approximately 20.12 and 26.94 Ma, respectively, compared with 11.9 Ma reported for maize and sorghum by Lai et al. [47]. Herendeen and Crane [48] published the fossil information regarding the Leguminosae family (51–60 Ma) from their infructescence organ. The mean Ks values of the 3 legume pairs *Glycine*–*Cajanus*, *Glycine*–*Medicago*, and *Cajanus*–*Medicago* were estimated to be 0.35, 0.42, and 0.37, with r values of 3.2 × 10^−9^, 3.9 × 10^−9^, and 3.4 × 10^−9^, respectively, with a calibration time of 54 Ma. The estimated divergence time of the legume plant, which was higher than that estimated by Lavin et al. [49] on the basis of maturase K and ribulose-1,5-bisphosphate carboxylase genes of the chloroplast. The closely related pairs *Glycine*–*Cajanus*, *Cajanus*–*Medicago*, and *Glycine*–*Medicago* were estimated to have diverged 23.88, 8.18, and 36.38 Ma, respectively. We used a calibration time of 400 Ma for the fungal species [50] and observed that *P*. *graminis* forms a monophyletic group with *C*. *gatti*, with a divergence time of 91.56 Ma. The fossil information revealed an evolution of wings in the insects approximately 315–300 Ma (http://www.kgs.ku.edu/Extension/fossils/insect.html). Peterson et al. [51] also reported the divergence of clade of tetrapod to be approximately 300 Ma. We used the maximum fossil calibration time of 315 Ma for estimating the divergence of fruit fly and mosquito; the average r value was estimated to be 0.77 × 10^−9^, with a median value of 0.23 × 10^−9^. We estimated that these 2 insect groups diverged from each other approximately 235.32 Ma. For analysing the divergence time in primates, we considered a fossil calibration time of 66 Ma [52]. Gorilla–orangutan and human–orangutan showed a close association with each other, with divergence times of 7.88 and 13.44 Ma, respectively (Table L and M in S2 File). Glazko and Nei [53] have estimated the divergence of human and orangutan during 12–15 Ma (13 Ma). In addition to the individual gene-based divergence analysis, we estimated the divergence times of the 49 species by using an uncorrelated lognormal relaxed-clock model and noted the origin of unicellular green algae *C*. *reinhardtii* to be nearly 1401.32 Ma. Furthermore, we estimated the origin of 2 model gymnosperm plants *P*. *taeda* and *P*. *glauca* to be approximately 261.82 Ma [95% highest posterior density (HPD): 250–285.34 Ma] in the middle of the Carboniferous period, which corresponds well with the reported fossil information [54] and a whole genome duplication [55]. We estimated the divergence time of angiosperms to be approximately 133.03 Ma (95% HPD: 130–138.97 Ma), which is close to the oldest reported fossil records of angiosperm (132 Ma) from the early Cretaceous period of the Mesozoic period. We sampled 9 fungal species for estimating the evolutionary distance and constructed a phylogenetic tree of life based on the conserved gene sequences among the 49 species to determine the fungal species more closely related to animals than to plants, as previously reported by Kuma et al. [56]. Furthermore, our analysis results suggest that fungi diverged from early life forms approximately 431.79 Ma (95% HPD: 415–467.04 Ma) during the Paleozoic era. In addition, invertebrate species diverged approximately 714.61 Ma (95% HPD: 700–745.19) in the late Proterozoic era. Similarly, vertebrates diverged from invertebrates approximately 340.669 Ma (95% HPD: 330–361.95 Ma).

RETRACTED

**Table 3:** Divergence times of 50 sampled pairs of species out of total 1,176 pairs of species anlysed (Table L in S2 File).

Organism Combination	Calibration Time (Ma)	Reference	Synonymous substitution rate based on mean Ks Value	Estimated Date in million years ago (Ma)
*O*. *sativa* vs. *Z*. *mays*	110	[35]	1.59E-09	53.46
*Z*. *mays* vs. *Sorgham bicolor*	110	[35]	1.04545E-09	31.73
*T*. *aestivum* vs. *Hordeum vulgare*	110	[35]	5.91E-10	42.37
*O*. *sativa* vs. *M*. *acuminata*	110	[35]	2.27273E-09	22.03
*O*. *sativa* vs. *B*. *distachyon*	110	[35]	1.54545E-09	61.69
*G*. *max* vs. *C*. *cajan*	54	[48]	3.24074E-09	24.55
*G*. *max* vs. *M*. *truncatula*	54	[48]	3.88889E-09	36.84
*C*. *cajan* vs. *M*. *truncatula*	54	[48]	3.42593E-09	7.35
*A*. *thaliana* vs. *V*. *vinifera*	100	[107]	3.4875E-09	29.89
*T*. *aestivum* vs. *A*. *thaliana*	200	[107]	1.40E-09	46.65
*P*. *taeda* vs. *P*. *glauca*	270	[108]	5.92E-10	49.92
*M*. *acuminata* vs. *P*. *taeda*	350	[55]	8.30E-10	35.84
*O*. *sativa* vs. *C*. *reinhardtii*	968	[16]	2.22E-10	180.18
*C*. *reinhardtii* vs. *P*. *patens*	1500	[109]	1.68E-10	515.57
*C*. *reinhardtii* vs. *D*. *discoideum*	1547	[110]	7.02E-11	209.76
*C*. *reinhardtii* vs. *P*. *infestans*	1642	[110]	1.38E-10	1117.52
*P*. *graminis* vs. *C*. *gattii*	400	[50]	6.3441E-10	91.56
*F*. *oxysporum* vs. *N*. *crassa*	400	[50]	4.95979E-10	93.95
*F*. *oxysporum* vs. *M*. *grisea*	400	[50]	4.81E-10	112.92
*M*. *grisea* vs. *A*. *oryzae*	400	[50]	5.87432E-10	96.42
*S*. *rosetta* vs. *C*. *elegans*	1538	[110]	1.76E-10	495.43
*A*. *oryzae* vs. *O*.*sativa*	1642	[110]	1.80E-10	586.59
*R*. *oryzae* vs. *T*. *aestivum*	1642	[110]	1.81E-10	439.64
*D*. *melanogaster* vs. *A*. *gambiae*	315	[111]	7.62E-10	235.26
*B*. *mori* vs. *S*. *purpuratus*	670	[112]	3.99E-10	143.26
*A*. *gambiae* vs. *C*. *reinhardtii*	700	[16]	3.51E-10	404.14
*D*. *melanogaster* vs. *M*. *Musculus*	964	[16]	2.82E-10	343.79
*B*. *mori* vs. *T*. *aestivum*	1547	[110]	1.87E-10	337.97
*C*. *elegans* vs. *S*. *purpuratus*	670	[112]	4.89E-10	182.72
*H*. *magnipapillata* vs. *N*. *vectensis*	741	[113]	1.60E-10	102.83
*C*. *intestinalis* vs. *H*. *magnipapillata*	1298	[16]	1.89E-10	174.34
*S*. *purpuratus* vs. *D*. *reio*	600	[112]	3.98E-10	124.23
*D*. *reio* vs. *X*. *laevis*	400	[113]	8.22E-10	103.89
*D*. *reio* vs. *G*. *gorilla*	445	[51]	6.42E-10	80.41
*D*. *reio* vs. *P*. *sinensis*	450	[114]	6.29E-10	105.92
*D*. *reio* vs. *D*. *melanogaster*	964	[16]	2.01E-10	308.96
*D*. *reio* vs. *P*. *abelii*	445	[51]	5.40E-10	60.81
*P*. *sinensis* vs. *A*. *caroliensis*	315	[115]	6.91E-10	101.48
*G*. *gallus* vs. *X*. *laevis*	350	[114]	7.52E-10	65.71
*X*. *laevis* vs. *A*. *caroliensis*	340	[116]	1.16E-09	68.65
*X*. *laevis* vs. *M*. *Musculus*	340	[116]	8.96E-10	95.81
*X*. *laevis* vs. *P*. *sinensis*	340	[116]	7.54E-10	84.48
*X*. *laevis* vs. *A*. *thaliana*	1547	[110]	1.85E-10	345.90
*P*. *sinensis* vs. *G*. *gallus*	340	[16]	7.54E-10	84.48
*G*. *gallus* vs. *M*. *Musculus*	300	[50]	7.75E-10	136.14
*G*. *gallus* vs. *B*. *mori*	964	[116]	2.74E-10	159.12
*P*. *abelii* vs. *H*. *sapiens*	66	[117]	8.49E-10	13.44
*B*. *tourus* vs. *T*. *gondii*	1547	[118]	1.62E-10	480.40
*O*. *sativa* vs. *H*. *sapiens*	1547	[110]	2.29E-10	545.85
*C*. *reinhardtii* vs. *H*. *sapiens*	1547	[110]	1.51E-10	820.67

RETRACTED

## Discussion

This study identified genes expressed uniquely in rice as well as those expressed commonly in diverse eukaryotic species—plants, animals, fungi, and protists. Such information can be studied further with an ultimate goal of crop improvement and establishing a platform for analysing evolutionary relationships among diverse taxa. The present study conducted a comprehensive genome-wide analysis of 49 model species representing diverse eukaryotic taxa. Of the 36002 expressed rice genes, 9831 unique rice genes are distributed in all 12 rice chromosomes. Of these unique genes, 64.21% (6313 genes) are TE-related; this emphasising the importance of repetitive elements in the evolution and expansion of the rice genome. The role of TEs in genome expansion and differentiation as well as the conservation of most functional genes has been well documented in rice, wheat, and maize with respect to their wild relative species [12, 57]. Furthermore, we could annotate 11.5% (1130 genes) of the unique rice genes with varying functions; however, the functions of the remaining 24.29% (2388 genes) remained unknown function, necessitating further characterisation. Among the annotated genes, most genes encoded F-box domain proteins that are essential during panicle and seed development in rice [58]. The second largest category of annotated unique rice genes comprised 122 genes for disease resistance and defence response-like proteins. The rice-specific disease resistance genes must have coevolved with obligate rice pathogens [59, 60]. Furthermore, 106 unique rice genes encoded for zinc finger proteins, which play a crucial role in stress tolerance [61]. Unique protein kinases, seed storage proteins as well as no apical meristem proteins was due to species-specific variations fixed in rice. Although these categories of genes have been reported in other cereals also but they can accommodate relatively large amounts of variations [62, 63].

The 9831 unique rice genes are crucial for maintaining rice as a distinct species with its unique biology and product value for human nutrition. By contrast, a large-scale homology-based data analysis of the 98 expressed rice gene homologues conserved in all 49 species revealed that this core set of genes is conserved among diverse eukaryotic species, including plants, animals, fungi, and protists. This is the largest number of species considered together for a genome-wide analysis of conserved genes. In 2007, Parra et al. [64] reported 248 core eukaryotic genes conserved in 26 species, which were a part of 4852 eukaryotic orthologous groups (KOGs) identified in 6 species [65] and 5873 KOGs in 7 eukaryotic species (*A*. *thaliana*, *C*. *elegans*, *D*. *melanogaster*, *H*. *sapiens*, *Saccharomyces cerevisiae*, *Schizosaccharomyces pombe*, and *Encephalitozoon cuniculi*) [66]. The total number of genes conserved across all the species decreases with the increasing number of species considered for comparison. The comparative analysis of exon and intron distribution revealed that the average number of exons is 4 in the unique rice genes and 7 in the genes conserved across species. Although the unique genes are on average smaller in size (3.04 kbp) compared with the conserved genes (4.00 kbp), their exon density (1.34 per kbp) is significantly lower than the conserved genes (1.73 per kbp), corroborating previous results that the accumulation of introns in evolutionarily conserved genes [67, 68]. In total 9831 genes were expressed uniquely in rice when we compared all the forty-nine eukaryotic species including plants, animals, fungi and protisa, but there were 9838 genes uniquely expressed in rice when we compared only the seventeen other plant species. The annotation of the additional seven genes revealed that six of these belonged to transposable elements, namely LOC_Os01g69020: unclassified retrotransposon protein, LOC_Os02g11665: unclassified transposon protein, LOC_Os08g12460: Ty3-gypsy retrotransposon protein, LOC_Os08g20500: unclassified retrotransposon protein, LOC_Os09g01120: Ty3-gypsy subclass, retrotransposon protein, LOC_Os12g43165: Ty3-gypsy subclass, retrotransposon protein, and the seventh one was LOC_Os09g38730: 26S protease regulatory subunit 6B. These seven genes while showing no homology with any of the seventeen plant species analysed, must have significant homology with one or more of the animal, fungi or protista species, indicating their ancient origins. Transposable elements play important role in the evolution and speciation through the exonisation and intronisation processes [69–71]. The analysis of the 2841 expressed rice gene homologues conserved in 17 plant species revealed that most of these genes support the basic cellular functions, such as the calcium/calmodulin dependent protein kinases involved in cellular signalling [72] and proteins related to ras, a member of small GTPases superfamily regulating signal transduction in eukaryotic species [73]. Furthermore, 761 and 910 rice gene homologues are conserved among 7 fungal and 20 animal species, respectively. Among all analysed species *Dictyostelium* showed the lowest level of homology with rice (n = 487), confirming the prediction of Eichinger and Noegel [74], who proposed that *Dictyostelium* is a suitable model organism for investigating conserved eukaryotic functions. Through pairwise genome comparison, we observed that 1056 of 53559 EST-unigenes of zebra fish (*D*. *rerio*), 988 of 34025 of chicken (*G*. *gallus*), 1222 of 70055 of human, and 1076 of 45364 of cow conserved in rice, respectively. According to these findings, thousands of proteins may be common between vegetarian (rice) and nonvegetarian (fish and chicken) sources of diet. In addition, conserved genes are not confined to rice chromosomes 1 and 3, although these 2 chromosomes possess the largest number of conserved genes having basic cellular function in all eukaryotic organisms; by contrast, chromosome 9 has the least number of conserved genes.

RETRACTED

The number of conserved rice gene homologues varies substantially, highlighting the process of origin and evolution of new genes. Most of the recently evolved or highly diversified unique rice genes are either TEs or those with unknown function. By contrast, the 98 ancient genes conserved across lower to higher eukaryotes have diverse known functions. A Bayesian phylogenetic tree of these 98 conserved rice genes can be grouped into 20 clades based on their common functions. These genes support extremely basic functions common to all eukaryotic species and must have originated at the dawn of the evolution of eukaryotes from their prokaryotic progenitors. Our most notable observation was that these genes have conserved sequence motifs among themselves, suggesting their common origin (Fig 6B). For instance, ADP-ribosylation and elongation factors having critical roles in protein translation in both prokaryotes and eukaryotes are clustered at the bottom of the tree along with DEAD-box proteinsthat alter RNA function [75]. Notably, ubiquitin, which is involved in proteosomal degradation [76, 77] and autophagy process conserved in all eukaryotic species [78], shares a common evolutionary node with tubulin, a homologous copy of which is also present in bacterial cells with filamenting temperature-sensitive mutant-z protein. Serine/threonine protein phosphatases, which play major roles in the biotic and abiotic stress responses [79, 80], are conserved from algae to human, form a clade along with casein kinase, which is biologically involved in the regulation of signal transduction pathways [43]. Our developed tree reveals the distribution and origin of different ubiquitin-mediated substrate degradation pathway-related proteins (26 protease and cell division control proteins).

RETRACTED

After analysing the biological functions and interrelationship of the 98 rice genes conserved across eukaryotes, we developed a eukaryotic tree of life based on the complete sequence information of these genes with no missing values. In 2007, Burki et al. [81] reported a tree of life based on 123 genes in 49 eukaryotic species but with 39% of missing data sets. Other studies have also reported trees of life, but based on limited number of genes (31 orthologous genes, [82]), or specific category of genes [83, 84], or single genes (e.g. small subunit of ribosomal RNA, [85]). However, the number of studies discussed the effect of missing data and their adverse impact on the incomplete fossil taxa [86–88] where as concatenated multigene data set logically reduces the noise of phylogenetic tree in comparison of single gene or few number of gene based phylogenetic tree [89, 90]. In the current scenario, a number of studies have addressed the issue of phylogenomics with the large pool of plant genome data sets using ML and Bayesian methodologies, for example Li et al. [91] reported 1469 single-copy genes conserved among 31 gymnosperm and 34 angiosperm plants, and appropriately highlighted the recent-ancestral divergence of seed plants. Similarly, Wickett et al. [92] have addressed the origin and evolution of land plants from their algal relatives using transcriptome data sets from 92 streptophyte taxa together with 11 plant genome sequence data. We developed both ML as well as Bayesian phylogenetic trees on the basis of the 98 gene sequences, but the level of nodal uncertainties was substantially high in the ML tree. For instance, among 7 fungal species, *R*. *oryzae* is more closer to the insects *A*. *mellifera* and *H*. *magnipapillata*, with a 94% bootstrap value. Similarly, *A*. *mellifera* is grouped with *C*. *interstinalis*, rather than the other 3 insect species (Figure K in S1 File). Bayesian posterior probabilities can quantify the uncertainty with regard to bootstrap values [93, 94]. Although previous studies have conducted bootstrap value-based analyses [95], we analysed a large data set, in which all eukaryotic species are grouped into 2 large clades of (i) plants and (ii) fungi and animals with a stable node support. All analysed protist species were included in 1 of these 2 clades. Among the 17 plant species, 5 Poaceae species are grouped in a single clade that evolved independently and is distantly related to the non-grassy plant banana. Our developed tree of life reveals the diversification of monocotyledonous and dicotyledonous plants, with banana establishing a link between the 2 clades. Furthermore, 20 animal species and 7 fungal species formed separate clades that are more closely related to each other than to the plant clade. Seven fungal species are grouped clearly in to the Ascomycota (*A*. *oryzae*, *F*. *oxysporum*, *N*. *crassa* and *M*. *grisea*), Basidiomycota (*P*. *graminis* and *C*. *gattii*), and Mucormycotina (*R*. *oryzae*). The strongly supported fungal species included Mucormycotina is ancestral, showing their link with protists. Among the 4 protist species, *D*. *discoideum* and *S*. *rosetta* are grouped with fungi and animal clades, respectively, whereas the 2 other species are closer to algal plants. The developed topology shows a diverse origin and association of protists with the 3 large groups of plant, fungal, and animal species. Our concatenated 98 conserved gene sequence-based Bayesian phylogenetic tree strongly supports the plant–protist–fungus and fungus–protist–animal groupings and rejects the theory of plant–animal grouping [96], based on the limited number of single family genes. The analysis of the 98 commonly expressed genes in the 49 model species reveals that the basic cellular machinery is composed of extremely similar proteins in all eukaryotes that strongly uniting plants, fungi, and animals with their protist allies; the species divergence is possible because of the large number of TEs and fast evolving species-specific functional genes [97].

RETRACTED

The **e**stimation of divergence times between species pairs is a crucial aspect of phylogenetic analyses. Here, we focused on the selection of appropriate statistical values for computing divergence times by using synonymous substitution (Ks) values and the corresponding mutation rate (r) for all 1176 pairs of analysed species. In earlier reports, divergence time been reported based on constant mutation rate in limited number of genes (e.g. in cereals r = 6.5 per site × 10^−9^ y have been used for the estimation of divergence time of different genes) [98, 99]. We estimated the average rate of synonymous substitution for every possible combination of genes among the 6 Poaceae family species, and the average synonymous substitution rate varied from 0.59 to 1.8 per site × 10^−9^ y for *Hordeum*–*Triticum* and *Sorghum*–*Brachypodium*. For the 7 dicotyledonous plant species the average r varied from 2.24 × 10^−9^ y for *Vitis–Populus* to 3.89 per site × 10^−9^ y for *Glycine–Medicago*; however, Koch et al. [100] reported r of 1.5 × 10^−8^ for dicotyledonous plants, differing considerably from 5.2 × 10^−9^ reported by Pfeil et al. [45], based on 39 genes of legume family. Among the 1176 pairs of species analysed here 15 pairs of species were from placental mammals, with estimated average r values of 0.58 per site × 10^−9^ y and 2.77 per site × 10^−9^ y for *Pan*–*Gorilla* and *Bos–Pan*, respectively. Li [101] estimated average Ks for mammals and *Drosophila* based on 47 and 33 protein sequences as 3.51 ± 1.01 per site × 10^−9^ y and 15.6 ± 5.5 per site × 10^−9^ y, respectively. These results may differ with the choice of genes as well as the number of genes used for analysis. The estimated r and divergence time of 1176 species pairs are valuable for future evolutionary divergence time-related studies. In general, we estimated the divergence times between species based on the Bayesian methodology. The 4 independent relaxed clock analyses with normal calibration priors highlight the evolution of different species and correspond well with the known fossil records. The combined log values suggest that the evolution time for the unicellular green alga *C*. *reinhardtii* is 1401 Ma, in the middle of the Proterozoic era (900–1600 Ma), which corresponds to the earliest known fossil records [33, 102]. Similarly, our Bayesian analysis results demonstrate that gymnosperms diverged in the early Permian period of the Paleozoic era (256–290 Ma), although Visscher et al. [103] and Foster and Afonin [104] have reported the presence of lycophyte spores and abnormal pollen grains of gymnosperms in the Permian-Triassic period approximately 252.53 Ma. Our analysis on the basis of a large data set yielded the divergence time for angiosperms to be the early Cretaceous period [105–106]. All analysed fungal species of Ascomycota, Basidiomycota, and Mucormycotina diverged in the middle of Ordovician period followed by Silurian and the early Devonian period of the Palaeozoic era. The vertebrate species diverged between late Devonian period to Mississippian Carboniferous period, whereas invertebrate species diverged in the late Proterozoic era. Notably, our genome-wide comparison and identification of 98 conserved genes among 49 diverse eukaryotic species provided most comprehensive and hence accurate basis for estimating the divergence times of plant, fungal, and animal species. The genome wide analysis of divergence time clearly highlights the evolution and divergence times of individual group of species. The use of different calibration times based on the relevant fossil records provides more accurate values than the use of a single calibration time for the entire spectrum of species.

RETRACTED

## Conclusions

Our genome-wide comparative analysis of a comprehensive set of expressed rice gene homologues in the 48 diverse eukaryotic species reveals information regarding the recently evolved rice-specific genes and the ancient genes conserved across eukaryotes. The presence of a common set of 98 conserved genes across diverse eukaryotic species underlined their role in the basic structural and metabolic functions and helped provide a clue regarding the origin and diversification of these species. A eukaryotic tree of life based on the comprehensive set of the conserved genes increases our understanding of the phylogenetic relationships among different plant, animal, fungal, and protist species. The grouping of protists within diverse clades emphasises their broad distribution and close association with the 3 eukaryotic clades—plants, animals, and fungi. In particular, *S*. *rosetta* provided a link between fungal and animal species, *T*. *gondii* provides a link between fungal and plant species, and *C*. *reinhardtii* is the nearest to the plant clade. The use of a comprehensive set of conserved gene sequences for estimating synonymous substitution rates and integration of fossil information provides more accurate estimation of the divergence time among a large number of species pairs by minimising the uncertainty associated with considering a small set of genes. This study provides novel information on the phylogenetic distances between some species pairs.

## Supporting information

S1 File **All supplementary figure information from A-K**.
**Figure A. Chromosome wise distribution of unique to rice gene.** (a) 9,831 expressed genes unique to rice (b) Proportion of the unique genes to total number of expressed rice gene.
**Figure B. Functional categorization of 9,831 genes uniquely expressed in rice.** Analysis progress graph shows number of matched with NCBI non-redundant (nr) as well as InterProScan database with mapping and annotation (a). All sequences have been categorized based on three GO (Gene Ontology) criteria namely biological function (b), cellular function (c) and molecular function (d) by BLAST2Go programme.
**Figure C. Distribution of conserved genes among 17 different plant species.** (a) Distribution of 57 large families (≥ 10 genes) of genes representing 1,871 of 2,841 genes conserved among 17 different plant species. (b) Chromosome wise distribution of 2,841 genes.
**Figure D. Chromosomal distribution of 313 expressed rice genes conserved in seven different fungal species**.
**Figure E. Categorization of conserved homologs rice gene in seven fungal species.** Annotation of 313 rice gene homologs conserved in seven fungal species grouped into 51 different families, of which 257 genes belonged to 19 major families each with more than five genes. Other 32 families have less than four copy of gene.
**Figure F. Distribution of 238 conserved rice gene homologs in four different protista species, namely *Phytophthora infestans*, *Salpingoeca rosetta*, *Dictyostelium discoideum* and *Toxoplasma gondii***.
**Figure G. Functional categorization of 238 conserved rice genes among four Protista species.** There were total 40 different functional categories, of which top 17 categories with more than five genes each, included 188 genes.
**Figure H. Functional categorization of 154 conserved rice genes among 20 different animal species (eleven vertebrate and nine invertebrate) into 30 different categories**.
**Figure I. Functional categorization of 727 conserved rice genes among six mammalian species.** There were total 156 different functional categories, of which top 35 categories each with more than five genes included 524 genes.
**Figure J. Motif prediction in conserved gene sequence.** Motif is generated in the 98 conserved gene sequence of the rice which has conserved among the 49 different eukaryotic organisms using MEME suite (Bailey and Gribskov 1998). Sequences has grouped into 22 different functional categories which shows the adequate conservation of motifs. Each block in the predicted motifs shows the location and height of the motif indicate about the significance of the individual sites. The motif sites shown on above line from positive strand while sites shown below from the negative strand.
**Figure K. Maximum likelihood based phylogenetic tree.** Phylogenetic analysis of 98 gene conserved among the 49 different eukaryotic species shows the grouping of different taxa. In ML tree all the bootstrap value for each node are indicated in figure.
(DOCX)

S2 File **All supplementary table information from A-M**.
**Table A.** Functional annotation of 9,831 genes uniquely expressed in rice and grouped in to 247 different gene families
**Table B.** Details of 9,831 rice genes expressed uniquely in rice
**Table C.** Distribution of 2,841 expressed homologous rice gene grouped into 444 gene families conserved among 17 plant species
**Table D.** Distribution of 195 conserved rice gene homologs across nine invertibrate (*C*. *intestinalis*, *A*. *mellifera*, *D*. *melanogaster*, *B*. *mori*, *A*. *gambiae*, *C*. *elegans*, *N*. *vectensis*, *H*. *magnipapillata*, *S*. *purpuratus*) species
**Table E.** Distribution of 24 rice gene homologs expressed uniquely in nine invertibrate (*C*. *intestinalis*, *A*. *mellifera*, *D*. *melanogaster*, *B*. *mori*, *A*. *gambiae*, *C*. *elegans*, *N*. *vectensis*, *H*. *magnipapillata*, *S*. *purpuratus*) species out of 20 animal species
**Table F.** Distribution of 413 conserved rice gene homologs across eleven vertibrate (*H*. *sapiens*, *P*. *troglodytes*, *G*. *gorilla*, *P*. *abelii*, *B*. *tourus*, *M*. *musculus*, *P*. *sinensis*, *A*. *caroliensis*, *D*. *reio*, *X laevis*, *G*. *gallus*) species
**Table G.** Functional annotation of 98 rice genes conserved across 49 eukaryotic species
**Table H.** Exon—intron distribution of 98 rice gene homologs conserved across 49 eukaryotic species
**Table I.** Summary of the samples of the substitution model parameters of 98 rice genes conserved across 49 eukaryotic species.Model parameter summaries over the independent runs (98geneOsa.nex.run1.p & 98geneOsa.nex.run2.p) after the burning of the initial 25% sample run. The different parameters like six reversible substituion rates ((r(A<->C), r(A<->G), r(A<->T), r(C<->G), r(C<->T), r(G<->T)), four stationary state frequencies (Pi (A), Pi (C), Pi (G), Pi (T)) and shape of the gamma distribution of rate variation across sites (alpha) used for this analysis. The Nst (general structure of the substitution model is determined by the Nst) value for the GTR (Generalised time-reversible) model was six. PSRF: Potential scale reduction factor, ESS: Estimated sample size
**Table J.** Summary of the samples of the substitution model parameters of 98 genes conserved in all eukaryotic 49 species (98×49 = 4,802). Model parameter summaries the concatenated genes over the two independent runs (98gene49Sps.nex.run1.p & 98gene49Sps.nex.run2.p) after the burning of the initial 25% sample run. The different parameters like six reversible substitution rates ((r(A<->C), r(A<->G), r(A<->T), r(C<->G), r(C<->T), r(G<->T)), four stationary state frequencies (Pi (A), Pi (C), Pi (G), Pi (T)) and shape of the gamma distribution of rate variation across sites (alpha) used for this analysis. The Nst (general structure of the substitution model is determined by the Nst) value for the GTR (Generalised time-reversible) model was six. The average ESS values above 200 ensured about the convergence of date. PSRF: Potential scale reduction factor, ESS: Estimated sample size
**Table K.** Synonymous substitution (Ks) values of 98 conserved genes in pair wise combinations of 49 eukaryotic species as estimated using DnaSp v5 programme. Among all 115,248 possible gene combinations Ks values were observed in only 86,362 combinaitons. Abbreviations for species A and B used from first letter of genus and another two letter from species. Abbreviation, Aor: *Aspergillus oryzae;* Fox: *Fusarium oxysporum;* Ncr: *Neurospora crassa;* Pgr: *Puccinia graminis;* Ror: *Rhizopus oryzae;* Sro: *Salpingoeca rosetta;* Mgr: *Magnaporthe grisea;* Cga: *Cryptococcus gattii;* Pin: *Phytophthora infestans;* Ath: *Arabidopsis thaliana;* Cca: *Cajanus cajan;* Gma: *Glycin max;* Mtr: *Medicago truncatula;* Ptr: *Populus trichocarpa;* Sly: *Solanum lycopersicum;* Vvi: *Vitis vinifera;* Bdi: *Brachypodium distachyon;* Osa: *Oryza sativa;* Zma: *Zea mays;* Tae: *Triticum aestivum;* Hvu: *Hordeum vulgare;* Sbi: *Sorgham bicolor;* Mac: *Musa acuminata;* Cre: *Chlamydomonas reinhardtii;* Ppa: *Physcomitrella patens;* Pta: *Pinus taeda;* Pgl: *Picea glauca;* Bto: *Bos tourus;* Has: *Homo sapiens;* Mmu: *Mus Musculus;* Ptr: *Pan troglodytes;* Ggo: *Gorilla gorilla;* Pab: *Pongo abelii;* Psi: *Pelodiscus sinensis;* Carolina: *Anolis caroliensis;* Dre: *Danio reio;* Xla: *Xenopus laevis;* Cin: *Ciona intestinalis;* Gga: *Gallus gallus;* Spu: *Strongylocentrotus purpuratus;* Ame: *Apis mellifera;* Dme: *Drosophila melanogaster;* Bmo: *Bombyx mori;* Aga: *Anopheles gambiae;* Cel: *Caenorhabditis elegans;* Nve: *Nematostella vectensis;* Hma: *Hydra magnipapillata;* Ddi: *Dictyostelium discoideum;* Tgo: *Toxoplasma gondii;*
**Table L.** Estimated divergence time between 1,176 pairs of species based on synonymous substitution (Ks) values for 54–98 conserved genes
**Table M.** Divergence time matrix among the 49 different species. The divergence time between the species showed in million years ago. Colour code showed the different group of organisms.
(XLSX)
